The article "Detection of Apical Dental Resorption Caused by Endodontic Infection in Mice Using Fluorescence and Bright-Field Microscopy" was published in 2023. Journal: Scanning.

# Detection of Apical Dental Resorption Caused by Endodontic Infection in Mice Using Fluorescence and Bright-Field Microscopy

**DOI:** 10.1155/2023/4619503

**Published:** 2023-04-17

**Authors:** Marcio Santos de Carvalho, Luciano Aparecido de Almeida-Junior, Yuri Jivago Silva Ribeiro, Maya Fernanda Manfrin Arnez, Raquel Assed Bezerra da Silva, Fabrício Kitazono de Carvalho, Francisco Wanderley Garcia Paula-Silva

**Affiliations:** Department of Pediatric Dentistry, School of Dentistry of Ribeirão Preto, University of São Paulo, Brazil

## Abstract

The aim of this study was to evaluate the sensitivity, specificity, and predictive values of the fluorescence microscopy method in the detection of apical dental reabsorption after induction of apical periodontitis in animal models. Forty-first molars of mice, aged 6 to 8 weeks, had their root canals exposed to the oral environment or were maintained healthy as controls (*n* = 20). After 14 and 42 days, mice were euthanized and tissues were collected for histological evaluation by means of bright field and fluorescence microscopy. The accuracy of fluorescence microscopy in identifying apical external dental resorption was investigated using a diagnostic validation test based on the sensitivity (S) and specificity (E) properties. Bright-field microscopy revealed a higher number of specimens with scores of 1 to 3 - absence of apical dental resorption (*n* = 29; 52%), while fluorescence microscopy revealed a higher number of specimens with scores of 4 to 6 - presence of apical dental resorption (*n* = 37; 66%). Out of 56 specimens, 26 were TP, 11 were FP, and 19 were TN. No FN result was observed. Fluorescence microscopy presented a sensitivity value of 1, similar to the bright-field method, while specificity was lower (0.633). The accuracy of the fluorescent method to detect apical dental resorption was 0.804. Fluorescence microscopy revealed a higher number of false positive apical dental resorption than bright-field microscopy. The detection of apical dental resorption was not impacted by the sensitivity of the method but by its specificity.

## 1. Introduction

Apical periodontitis is the result of a localized immunoinflammatory response resulting from a persistent infectious process caused by the colonization of microorganisms within the dental root canal [1–3]. The composition of the endodontic microbiota includes several pathogenic microorganisms that trigger an innate and adaptive immune and inflammatory response mediated by various metabolites [1, 2, 4, 5]. This process is complex and results in extensive destruction of the periodontal ligament and mineralized tissues such as alveolar bone and dental root cementum, which may be associated with clinical manifestations and radiographic and histopathological findings [6, 7].

The article "Detection of Apical Dental Resorption Caused by Endodontic Infection in Mice Using Fluorescence and Bright-Field Microscopy" was published in 2023. Journal: Scanning.

To perform the histopathological and morphometric study of tissue changes in apical periodontitis, the bright-field microscopy method has been considered the gold standard to identify and measure the resorption of mineralized tissues in animal models [8–10]. Evaluation of tissue changes is performed through histotechnical processing; histological sections of mineralized tissues are stained with hematoxylin and eosin (HE) substances capable of highlighting the cell and morphological structures of healthy or pathologically altered tissues [11–13]. Bright-field and fluorescence microscopy allow the visualization of the tissue to identify the presence or absence of bone resorption [11, 12].

Morphometric analysis by fluorescence microscopy is a useful tool for the histological evaluation of mineralized tissues [12, 14]. In apical periodontitis, morphometric fluorescence analysis is used to evaluate the disorganization of the periodontal ligament and areas of resorption of the alveolar bone and dental root cementum [12]. In bone tissue, fluorescence microscopy improves the visualization of the periapical region, and the resorption areas become evident, being a reliable method for the quantitative study of bone loss in apical periodontitis [12, 14]. However, the reliability of the method to identify apical dental resorptions in the animal model is not known. Therefore, it is necessary to perform the diagnostic validation tests, using the histological method by bright-field microscopy as the gold standard.

In view of the above, this study is aimed at evaluating the sensitivity, specificity, and predictive values of the fluorescence microscopy method in the diagnosis of apical dental resorption after induction of apical periodontitis in mice.

## 2. Materials and Methods

### 2.1. Animals

This study was approved by the Animal Research Ethics Committee at the School of Dentistry of Ribeirão Preto, University of São Paulo, Brazil (process # 2021.1.280.58.8). Forty C57BL/6 male mice, aged 6 to 8 weeks, weighing 20 to 22 g, were used for experimentation.

### 2.2. Operative Procedures

Apical periodontitis was induced as previously described [15]. The animals were anesthetized intramuscularly with ketamine hydrochloride (150 mg/kg of body weight) (10% ketamine, Agener União Química Farmacêutica Nacional S/A, Embu-Guaçu/SP, Brazil) and xylazine (10 mg/kg of body weight) (2% xylazine, Dopaser, Laboratórios Calier S/A, Barcelona, Spain). To induce apical periodontitis, 1/4 spherical burs (KG Sorensen, Barueri/SP, Brazil) mounted in a high rotation pen (odontological equipment Dabi Atlante, Ribeirão Preto/SP, Brazil) were used to perform the occlusal coronary opening of the first lower molars. The root canals were left open to the oral environment for 14 and 42 days (*n* = 20 teeth per group). The contralateral molars were maintained healthy to evaluate apical dental morphology in teeth without root resorption (*n* = 20 teeth). After the experimental period, animals were euthanized using anesthesia followed by CO_2_ inhalation in a chamber.

The article "Detection of Apical Dental Resorption Caused by Endodontic Infection in Mice Using Fluorescence and Bright-Field Microscopy" was published in 2023. Journal: Scanning.

### 2.3. Histological Processing

During the histological processing, 4 teeth were lost, and histological analysis was done in 56 specimens. Then, histological cuts stained by hematoxylin and eosin (HE) were evaluated using bright-field microscopy (Zeiss Axiolab 5 Carl Zeiss AG light Microscopy, Göttingen, Germany). Fluorescence mode (Alexa Fluor filter 488-AF488, G365 excitation, FT395 reflectors, and LP420 emission) was used to evaluate the apical dental resorption, as previously described [12, 15, 16].

### 2.4. Evaluation of the Accuracy of Morphometric Fluorescence Analysis to Identify Apical Dental Resorptions

Using a diagnostic validation test based on the sensitivity (S) and specificity (E) properties, the accuracy of fluorescence morphometric analysis in identifying apical dental resorption was investigated. Bright-field microscopy was used as the gold standard. Individual values of positive and/or negative cases were calculated according to the dental resorption parameter using an ordinal evaluation scale: (1) definitely negative, (2) probably negative, (3) possibly negative, (4) possibly positive, (5) probably positive, and (6) definitely positive [17]. Scores from 1 to 3 were grouped as absence of apical dental resorption, while scores from 4 to 6 were grouped as presence of apical dental resorption. Based on the diagnosis on the bright field, the test was classified as true-positive (TV), true-negative (TN), false-positive (FP), and false-negative (FN). From the values obtained for sensitivity and specificity, a receiver operator characteristic (ROC) curve was done to determine the accuracy of the method [18]. To generate the ROC curve, all the values were ranked, and each value was linked to the diagnosis—absence of apical dental resorption (scores 1 to 3) and presence of apical dental resorption (scores 4 to 6).

## 3. Results

Bright-field microscopy revealed a higher number of specimens with scores of 1 to 3—absence of apical dental resorption (*n* = 29; 52%), while fluorescence microscopy revealed a higher number of specimens with scores of 4 to 6—presence of apical dental resorption 37 (66%) (Table 1).  Table 2 summarizes the results of the positive and/or negative diagnostic tests (TP, FP, TN, and FN) using the fluorescence method to detect apical dental resorption compared to bright-field microscopy. A total of 37 (66%) specimens showed apical dental resorption and 19 (34%) did not. Out of 56 specimens, 26 were TP, 11 were FP, and 19 were TN (Table 2). No FN result was detected. The sensitivity and specificity of the fluorescent method to detect apical dental resorption were calculated. Fluorescence microscopy presented a sensitivity value of 1, similar to the bright-field method, while specificity was lower (0.633). Accuracy of the fluorescent method to detect apical dental resorption was 0.804 (Figures 1 and 2).

The article "Detection of Apical Dental Resorption Caused by Endodontic Infection in Mice Using Fluorescence and Bright-Field Microscopy" was published in 2023. Journal: Scanning.

## 4. Discussion

It is known that inflammation and periapical bone resorption, in most cases, is a consequence of the interaction between the agent microbial inside the root canals and the host response [19]. And one of the characteristic findings of the apical periodontitis is the increasing recruitment and formation of osteoclasts in areas of active bone resorption [20]. Histopathological findings demonstrate that the operative procedure used in the current study induces apical periodontitis formation in murine teeth, as previously demonstrated by other researchers [2, 15, 21, 22].

Microscopic analysis, by means of bright-field microscopy and fluorescence methods, can be used to evaluate bone and apical dental resorption. Nonetheless, validation of these methods is fundamental to assess this parameter with accuracy and reliability [23]. Bright-field microscopy is considered the gold standard for the detection of the presence or absence of inflammatory infiltrate and bone and dental root resorption [8, 24]. Previous studies also showed that fluorescence allows a better identification and observation of the perimeter of apical periodontitis in the areas of bone resorption [2, 12, 14], opening the avenue for using this method to investigate the extent of apical dental resorption.

We found that fluorescence microscopy presents good accuracy (0.804) and sensitivity (1) to detect apical periodontitis. However, compared to bright-field microscopy, fluorescence microscopy shows low specificity (0.63) resulting in false-positive results during apical dental resorption detection. Previously, De Rossi et al. [12] stated that fluorescence microscopy enhances the visualization of the apical and periapical structures in periapical disease. However, for apical dental resorptions, we observed here that fluorescence showed dental resorptions in areas of health cementum thereby enhancing the number of false positive results. To the best of our knowledge, this is the first study to investigate the sensitivity, specificity, and accuracy of the fluorescence method in the diagnosis of apical dental resorption compared to bright-field microscopy.

The article "Detection of Apical Dental Resorption Caused by Endodontic Infection in Mice Using Fluorescence and Bright-Field Microscopy" was published in 2023. Journal: Scanning.

## 5. Conclusion

Fluorescence microscopy revealed a higher number of false positive apical dental resorption than bright-field microscopy. Detection of apical dental resorption was not impacted by the sensitivity of the method but by its specificity.

## Figures and Tables

**Figure 1:** ROC curve for the fluorescence method applied to identify apical dental resorption showing specificity and sensitivity with line inclination at 45°, indicating diagnostic accuracy.

**Figure 2:** Photomicrography of the distal root of the first molar of mice. (a, b) Bright-field and fluorescence microscopy: healthy tooth showing periodontal ligament, alveolar bone, dentin, and cementum. In both 14-day period (c, d) and 42-day period (e, f), dental resorption was observed in fluorescence (original magnification = 10x; scale bar = 100 *μ*m).

**Table 1:** Detection of the presence and absence of apical dental resorption using scores by means of bright field and fluorescence microscopic evaluation methods.

Parameter	Method	Score						Total
		(1)	(2)	(3)	(4)	(5)	(6)	
Apical dental resorption	Bright-field microscopy	14	4	11	16	4	7	56
	Fluorescence microscopy	8	3	8	14	10	13	56

**Table 2:** True-positive, true-negative, false-positive, and false-negative values in the detection of apical dental reabsorption by the fluorescence method.

Parameter	Method	Positive	Negative	TP	FP	TN	FN	Total
Apical dental resorption	Fluorescence microscopy	37	19	26	11	19	0	56

## Data Availability

The data used to support the findings of this study are included within the article.
